This article has been retracted.

# Income Uncertainty and Consumer Demand among Rural Residents Analysis Based on Optimisation of Household Consumption Utility

**DOI:** 10.1155/2022/2068963

**Published:** 2022-10-08

**Authors:** Xiejun Cheng, Yang Qiao, Qi Feng, Shenghua Huang

**Affiliations:** ^1^School of Business, Jiangsu Second Normal University, Nanjing, 211200 Jiangsu, China; ^2^School of Economics, Beijing Technology and Business University, Beijing, 100048 Beijing, China

## Abstract

As China enters a new era, the role of consumption as a driving force for the economy has become increasingly prominent. The consumption of rural residents is not only a matter of high-quality economic development but also an important part of realizing people's aspirations for a better life. This study contributes to the literature by establishing an econometric model based on the construction of a theoretical model for optimizing the utility of household consumption, using panel data from China's 31 provinces, eliminating endogenesis by using instrumental variables, taking  2*SLS* and dynamic  *GMM*. The results show that the relationship between income uncertainty and rural residents' consumption varies in the same direction, stimulating consumption when real income exceeds psychological income and reducing consumption when real income does not reach psychological income. The quantile model shows that income uncertainty has a greater impact on the middle-high-consumption groups and a smaller impact on the lower-income groups.

## 1. Literature Review

As one of the “troika” of economic growth in the traditional sense, the lack of demand for residential consumption is an important reason for the lack of pulling power for the economy. Therefore, the importance of residential consumption in social and economic development has become more prominent. The “14th Five-Year Plan” and the “visionary goal for 2035” clearly put forward “to build a new development pattern with the domestic circulation as the main body and the domestic and international circulation promoting each other,” with the domestic circulation as the main body means that we must expand and increase domestic demand. The main body of the domestic cycle means that it is necessary to expand domestic demand, increase the development of the domestic consumer market, meet the demand for upgrading domestic consumption, and provide a constant source of power for high-quality economic development. Rural residents, who account for nearly half of China's population, should not be neglected in terms of their consumption power on economic and social development, especially the huge consumption potential of rural residents. The “No. 1 Document” of the Chinese Central Government in 2021 focused on rural revitalization, proposing that “the whole party should make efforts to make the majority of farmers lead a better life” and explicitly requesting “to comprehensively promote rural consumption.” Subsequently, the National Rural Revitalization Bureau was established, and the Law of the People's Republic of China on Promoting Rural Revitalization was officially implemented. Therefore, how to effectively increase the income of rural residents and stimulate their consumption is a matter of overall economic development and an important element in building a happy China, realizing the “Chinese dream,” realizing people's aspiration for a better life and accomplishing the goal of “two hundred years.”

The research literature related to rural residents' income and consumption can be said to be overwhelming and innumerable, but the vast majority of studies are based on the perspective of income distribution and total income to study the impact of income on consumption ([1–9], etc). Some scholars also discuss it from the perspective of income composition, mainly dividing rural residents' income into persistent income and temporary income, with persistent income being more stable and expected income, which is the main source of supporting consumption, so persistent income is the main influence of rural residents' consumption vulnerable to loss, while temporary income is unstable and does not enable consumers to generate future income expectations.

The influence effect on consumption is weak, while studies also find that the marginal propensity to consume is greater for persistent income and smaller for temporary income ([10–12], etc). At the same time, relative to Chinese urban residents, the growth rate of rural residents' persistent income is relatively slow and vulnerable to external environmental factors, e.g., the returns of crops are vulnerable to the natural environment and market supply and demand, and there is a certain degree of uncertainty, while the uncertainty of temporary income is even stronger and the marginal propensity to consume is already small, thus causing the overall marginal propensity to consume of rural residents to be smaller.

In the early days of the dualistic household registration system, the main source of income for farmers came from net business income, while other types of income were negligible. With the loosening of the household registration system and the increasing scale of population mobility, the number and proportion of rural residents moving to the cities for work have been rising, resulting in a marked increase in farmers' wage income; in recent years, along with the increasing attention paid by the state to the “three rural issues” and the gradual opening of land transfer, farmers' net property income and net transfer income have also been increasing. The impact of different sources of income on consumption has also changed accordingly, which has attracted the interest of some scholars.

For rural residents, the share of net business income in total income has been declining in recent years in general, but the total amount is increasing, and it is a relatively large and stable source of income, which plays a very obvious role in supporting basic consumption [13, 14]. The rapid development of urbanization has increased a large number of non- agricultural employment opportunities for rural residents, and the continuous improvement of transportation and other basic facilities has provided a good basis for rural residents to work in cities, the wage income of rural residents has grown faster, the growth rate has been higher than that of net business income since 2000, and the influence on rural residents' consumption has gradually increased [15]. The net property income of rural residents mainly comes from land, houses, and idle capital; the value of houses in rural areas is not high, farmers have less idle capital due to income constraints, and the transfer fees for land are not high, resulting in a relatively low level of net property income all the time despite the growth, which ultimately makes the consumption effect of net property income limited, mainly in the promotion of food consumption [16–18]. With the improvement of the level of social security and basic public services in rural areas, the increase in government financial expenditure on education has also alleviated the education expenditure of rural residents' children, and the net transfer income received by rural residents is growing, which has a positive effect on promoting consumption, but as the absolute value is still at a low level, the impact on rural residents in some areas is not yet significant [19].

Many factors affect the income of rural residents, among which there are also highly contingent and unpredictable factors, such as weather, natural disasters, market prices, and policy preferences, leading to a high level of uncertainty about rural residents' income, which has a significant impact on their consumption [20–23], and an increase in uncertainty can influence consumption behavior towards caution to the extent that it reduces consumption and increases savings [24–27]. With China's rapid socioeconomic development, the uncertainties affecting rural residents' income are also increasing, and the negative impact of income uncertainty on rural residents' consumption is significantly higher than that of urban residents due to the motive of precautionary saving and the sensitivity of consumption to income [28–32].

The literature is a good reference for clarifying the factors affecting consumption and the relationship between consumption and income. Most of the studies have explained how the changes in consumption are affected from the perspectives of consumption habits, total income level, fiscal expenditure, and public goods. The relationship between income level or income level and consumption has also been adequately studied, and the empirical studies have mainly adopted time series and panel. The empirical studies have mainly used time series and panel data analysis methods. However, after careful examination, it is found that there are still areas that need to be added.

For example, the impact of income uncertainty on consumption demand is mainly at the level of normative analysis, but not much quantitative analysis is available. The reliability of the findings is debatable.

Drawing on existing studies, this paper attempts to make up for the above shortcomings, with the following possible academic marginal contributions: using two methods to measure income uncertainty, paying particular attention to reflecting the directionality of income uncertainty through the choice of measurement method, this is a clear departure from most of the current research; paying attention to analyzing the positive impact that income uncertainty may play on consumption when constructing a consumer utility maximization model changes the existing research often pays attention to the negative influence which the income uncertainty plays, ignores the possible positive influence, enriches the research to this question, and then conducts a comparative analysis on the basis of the overall study by time period. The model was constructed with attention to the possible positive impact of income uncertainty on consumption, and on the basis of the overall study, two types of econometric analyses were carried out: time period and subregion, and a comparative regression analysis was conducted using different income uncertainty indicators to enhance the stability and reliability of the empirical findings as far as possible.

## 2. Theoretical Model Construction

It is assumed that the principle of representative rural household consumption is utility optimisation, i.e., *u* = *u*(*c*), where *u* denotes utility and *c* denotes consumption.

Given the temporal inconsistency between income and consumption, consumers tend to base their consumption on earned income, i.e., consumption is often influenced by income from the previous period rather than the current period; current consumption is influenced by past consumption habits due to the “ratchet effect”; optimistic future income expectations will boost current consumption, and pessimism will discourage it; the price level of consumer goods will also have a significant impact on consumers, i.e., the current price level will influence consumption demand; with urbanization, the income level and structure of the rural population will influence consumption demand to a large extent. The price level of consumer goods also has a significant impact on consumers, i.e., the current price level affects consumer demand; as urbanization progresses, the income level and structure of rural residents have changed significantly, which also affects consumer demand. In addition to this, factors such as policies and consumer preferences can also have different effects. Combined with the research objectives of the article, it is assumed that the factors affecting representative household consumption are income level, consumption habits, income uncertainty (the uncertainty of income is used here in place of future income expectations, and the specific measurement is described below.), price level, and urbanization rate, and the effects of other factors (such as policy and social security level) are represented by random error terms. The above utility function is therefore deformed as follows:

(1) $$\begin{array}{c} u_{t}=u\left(c_{t-1},y_{t-1},y_{t}^{i},p_{t}\right). \end{array}$$

In Equation (1), *c*_*t*−1_ represents past consumption habits, *y*_*t*−1_ represents prior period income, *y*_*t*_^*i*^ represents income uncertainty, and *p*_*t*_ represents current price levels.

The relatively low level of income and uncertainty of rural households leads to a tendency for rural households to be conservative in their consumption, so the utility function of rural households can be assumed to be constant absolute risk aversion function (CARA) and Equation (1) can be replaced by

(2) $$\begin{array}{c} u_{t}=-\frac{1}{\theta }\exp\left\{-\theta \left(\alpha_{1}c_{t-1}+\alpha_{2}y_{t-1}+\alpha_{3}y_{t}^{i}+\alpha_{4}p_{t}\right)\right\}, \end{array}$$

where *θ* is the absolute risk aversion coefficient and *α* is the parameter for each variable.

Households face a budget constraint when making consumption decisions, and since real estate such as the rural household home is not easy to realize, household income is considered the only constraint. The constraint is then

(3) $$\begin{array}{c} \sum p_{t}c_{t}=y_{t-1}. \end{array}$$

Therefore, the representative household utility optimization can be expressed as

(4) $$\begin{array}{c} \max\left\{-\frac{1}{\theta }\exp\left[-\theta \left(\alpha_{1}c_{t-1}+\alpha_{2}y_{t-1}+\alpha_{3}y_{t}^{i}+\alpha_{4}p_{t}\right)\right]\right\}. \end{array}$$

The constraint is Equation (3).

## 3. Measurement of Revenue Uncertainty

There are about three types of measures of income uncertainty: first, the proxy variable approach, which uses economic indicators that have some correlation with income uncertainty as a proxy, such as the unemployment rate, economic growth rate, standard deviation, or variance of income groupings, and the difference between trend and actual values of income ([33–36], etc). The second is the questionnaire method, i.e., the subjective evaluation of respondents is obtained through questionnaires, and uncertainty is obtained through statistical analysis [37]. The third is the use of adjusted deviation rates to calculate income uncertainty [38–40].

Proxy variables can explain income uncertainty to different degrees and are indirect measures of income uncertainty, which have the shortcoming of being too homogeneous and can only reflect income uncertainty from one aspect, resulting in large differences between the findings of different proxy variables, and are not reliable enough. Questionnaire surveys can avoid the indirectness of proxy variables and directly calculate income uncertainty, but the questionnaire design lacks uniform specifications and relies on the designer's perception of income uncertainty, which is relatively weak in objectivity, in addition to not being able to obtain continuous data and cannot conduct dynamic research. According to Knight's (1921) definition of uncertainty, income uncertainty should be the fluctuation of income that are not within the range of public expectation, i.e., it should be equal to the difference between expected income and actual income. Uncertainty itself should be directional, with positive values having a positive effect on consumption, i.e., a “windfall” stimulating consumption, and negative values having a negative effect, i.e., a “loss of income” inhibiting consumption. Adjusting for deviations reflects both the degree of deviation between unanticipated and actual income and is suitable for continuous data. For these reasons, this paper uses two methods to measure income uncertainty: the first is to choose the adjusted deviation rate used by Wang et al. to measure income uncertainty, and the second is to use the HP filter to isolate fluctuations in the actual income of rural residents and use the fluctuate on value as an indicator of income uncertainty. The empirical part uses the data from the above two measures separately for empirical analysis and comparison to make the findings more reliable.

Assuming that the actual income of rural residents in year *t* is *y*_*t*_, the expected income is *y*_*t*_^*e*^, the annual income growth rate that rural residents can expect is *k*_*t*_%(*k*_*t*_% taking the arithmetic average of the real income growth rate of rural residents in every three years), and the real income growth rate in year *r*_*t*_% is denoted as

(5) $$\begin{array}{c} y_{t+1}^{e}=y_{t}\left(1+k_{t+1}\%\right),\\ k_{t+1}\%=\frac{r_{t-2}\%+r_{t-1}\%+r_{t}\%}{3}. \end{array}$$

From Equations (1) and (2), the expected income of rural residents in each year can be calculated, and the adjusted deviation in the first *t* years is

(6) $$\begin{array}{c} {AD}_{t}=y_{t}^{e}-y_{t}. \end{array}$$

Further, due to factors such as price increases and income levels, the adjustment deviations between periods cannot be compared only in absolute magnitude, and the uncertainty of income can be better expressed by using the ratio of adjustment deviation to actual income, noted as *EAD*_*t*_ as the adjustment deviation rate in *t* years, with

(7) $$\begin{array}{c} {EAD}_{t}=\frac{{AD}_{t}}{y_{t}^{e}}\times 100\%=\frac{y_{t}^{e}-y_{t}}{y_{t}^{e}}\times 100\%=1-\frac{y_{t}}{y_{t-1}\left(1+k_{t}\%\right)}\times 100\%. \end{array}$$

The positive and negative signs of the adjusted deviation rate calculated according to Equation (7) represent the direction of income uncertainty, *EAD*_*t*_ > 0, indicating that rural residents are overoptimistic about their future income and their actual income does not reach their expected income, resulting in an “income loss”; *EAD*_*t*_ < 0 indicating that rural residents' actual income exceeds their expected income, resulting in a “windfall.” The negative sign represents the direction of income uncertainty.

## 4. Empirical Results and Interpretation

### 4.1. Description of Data and Variables

The original data used in this paper are all from China Statistical Yearbook and Wind database, except the price index, and the other indicators are per capita level, all of which exclude the price factor to be comparable data.

#### 4.1.1. Explained Variables

In per capita consumption level *RC*_*t*_, according to the National Bureau of Statistics of the People's Republic of China's interpretation of household consumption expenditure, household consumption expenditure includes cash consumption expenditure and in kind consumption expenditure, so we use a unified indicator of household consumption expenditure to measure the per capita consumption level.

#### 4.1.2. Core Explanatory Variables

In income uncertainty, the expected income of consumers will affect consumption, the expected income is the subjective judgment of future income, and the actual income often has a certain margin, so we can use the income uncertainty to replace. Based on the analysis in Section 3, this is measured using *EAD*_*t*_ or income fluctuations ln*Y*_*tv*_ (obtained using the *HP* filter method).

#### 4.1.3. Control Variables

In per capita income level *RY*_*t*_, according to the change of the statistical caliber of the National Bureau of Statistics, the income indicator of rural residents was changed from net income per capita to disposable income per capita (used since 2013, due to the unified implementation of the household income and expenditure and living conditions survey system from 2013), in order to ensure the consistency of the data, the data were processed with the base period of 1998, and the indicator of disposable income per capita was used uniformly to measure.

In price level *P*_*t*_, as the study is on the consumption level of rural residents, the Consumer Price Index for Rural Residents is used as a measure.

In urbanization rate *UR*_*t*_, it is expressed using the number of urban population as a proportion of the total population.

Taking into account the large differences between East, Central, and West China, regional dummy variables *A*_1_ and *A*_2_ are introduced, defined as *A* value of *A*_1_ is 1 for the eastern region and 0 for the other regions; a value of *A*_2_ is 1 for the central region and 0 for the other regions.

In order to eliminate possible heteroscedasticity and skewness and reduce the influence of extreme values on the model, natural logarithmization was done for the above variables except dummy variables. Taking into account the availability and consistency of data to ensure sufficient observations, this paper selects annual data from 31 provinces (municipalities and autonomous regions) throughout the country from 2000 to 2020, Hong Kong, Macao, and Taiwan are not included.

### 4.2. Econometric Model Construction

Based on the above analysis, and considering that consumption is generally influenced by prior period income, rather than current period income, the econometric model constructed in this paper is

(8) $$\begin{array}{c} \ln{RC}_{t}=\alpha_{0}+\alpha_{1}\ln{RC}_{t-1}+\alpha_{2}\ln{RY}_{t-1}+\beta \ln{EAD}_{t}+\delta_{1}\ln p_{t}+\delta_{2}\ln{UR}_{t}+\overset{2}{\underset{i=1}{\sum }}\lambda_{i}Ai+\varepsilon , \end{array}$$

(9) $$\begin{array}{c} \ln{RC}_{t}=\alpha_{0}+\alpha_{1}\ln{RC}_{t-1}+\alpha_{2}\ln{RY}_{t-1}+\beta \ln Y_{tv}+\delta_{1}\ln P_{t}+\delta_{2}\ln{UR}_{t}+\overset{2}{\underset{i=1}{\sum }}\lambda_{i}Ai+\varepsilon . \end{array}$$

A comparative analysis of model (8) and model (9) allows testing whether different measures of income uncertainty affect the reliability of the conclusions.

Based on the use of Chinese subprovincial data, the impact of income structure and its uncertainty on consumption will be empirically analyzed in three stages, with the first stage focusing on testing the smoothness and cointegration of the variables, the second stage selecting the most appropriate model form through testing, and the third stage testing the stability of the model, including a discussion of issues such as endogeneity, and analyzing the impact of income uncertainty at different levels of consumption through a quantile model impact changes.

### 4.3. Empirical Results

#### 4.3.1. Descriptive Statistics for Variable Data

In order to better understand the characteristics of the numerical values of the variables, descriptive statistics of the variables and statistical analysis of the results are shown in Table 1.

Table 1 shows that the mean and median values of the variables are close to each other, indicating a regular distribution of the values of the variables. The largest difference between the maximum and minimum of each variable is the level of per capita consumption, indicating that per capita consumption is more volatile than other variables and that the maximum and minimum of income uncertainty are quite different; it shows that the change of rural residents' income in China is also quite obvious. The corresponding standard deviation of each variable also confirms the above conclusion. If the standard deviation of average consumption level is the largest, it also shows that its volatility is the largest. The skewness value shows that the income uncertainty expressed by the adjusted interest rate is a left-skew distribution, per capita consumption level, per capita income level, urbanization rate, price level, and income uncertainty expressed by income fluctuation which are right skew distribution. Since the peak value of all variables is greater than 0, the distribution of the values of each variable is steeper than that of the normal distribution and is the peak, especially when the peak value of income uncertainty is greater than 3, indicating a very steep distribution, the peak value of other variables is less than 3, which indicates that the steepness is limited. The J-B statistics of each variable also verifies the skewness value and the analysis results.

#### 4.3.2. Unit Root Test for Panel Data

To avoid possible bias in the estimation results caused by each variable not being a smooth series, two methods with opposite assumptions are used for testing, an *LLC* method that assumes all cross-sections have the same unit root and an *ADF* method that assumes all cross-sections have different unit roots. The test results are shown in Table 2.

The above test results show that the *LLC* test and *ADF* test of the original series of ln*RC*_*t*_, ln*RY*_*t*_, ln*UR*_*t*_, ln*P*_*t*_, ln*EAD*_*t*_, and ln*Y*_*tv*_ show a nonstationary series, the first-order difference series of 1 shows a first-order stationary series except ln*Y*_*tv*_, and the *PP* test of ln*Y*_*tv*_ shows a first-order stationary series. Therefore, the above variables are homogeneous single-integer series, and theoretically, there is cointegration relationship.

#### 4.3.3. Cointegration Test of Panel Data

Each variable is a single-integer sequence of the same order, and the cointegration test is used to test whether there is a long-term equilibrium relationship. The test results are shown in Tables 3 and 4.

The above results show that the variables in Equations (8) and (9) reject the “original hypothesis of no cointegration relationship” except for the within-group *v* − *Stat*, *rho* − *Stat*, and between-group *rho* − *Stat* statistics, and the overall judgment is that there is a cointegration relationship between the above panel variables.

## 5. Estimated Results

### 5.1. General Panel Regression Results

The variables used are cointegrated and can be regressed. The model was first estimated using least squares (5) and was found to be potentially autocorrelated, with coefficient tests on the regional dummy variables showing that none were significant (regression results omitted). To determine the appropriate panel model type, the *F* test and *Hausman* test were used to determine the model category, with the *F* test used to determine whether to build a mixed model or a fixed-effects model and the *Hausman* test used to determine whether to build a fixed-effects model or a random-effects model. The value of the *F* test is calculated as 45.271, rejecting the original hypothesis that the true model is a mixed model and accepting the fixed-effects model, while the value of *P* for the *Hausman* test is 1.000, indicating that the original hypothesis of “the random-effects model is valid” is accepted at both 5% and 10% significance levels. For this reason, the panel random-effects model is chosen, and the estimation results of the fixed-effects model are also given for comparison. The estimate is shown in Table 5.

The results of the random-effects estimation are in full agreement with the fixed-effects estimation, the goodness of fit reaches 99.5%, the *F* test passes, and the *D* − *W* values can basically exclude autocorrelation and the regression results are acceptable without considering endogeneity. The results show that the per capita income in the previous period, urbanization, price level, income uncertainty, and per capita consumption in the previous period are all positively correlated with per capita consumption.

It is worth noting that the coefficient of income uncertainty is positive, i.e., income uncertainty moves in the same direction as consumption, but it does not mean that income uncertainty will necessarily boost rural residents' consumption; it is important to note that there are positive and negative income uncertainties calculated above. When income uncertainty is negative, it means that rural residents have lost their expected level of income and their consumption sentiment tends to be pessimistic, favouring increased saving as opposed to consumption. Both cases are consistent with a homogeneous relationship between the two, but the positive and negative results affecting rural residents' consumption are different, which is quite different from the existing literature which mostly considers that income uncertainty has a negative impact on consumption. In addition, by regressing the uncertainty of per capita consumption and income and its quadratic term, it is found that the estimated coefficient of quadratic term is positive, which means that there is a U-shaped relationship between per capita consumption and income uncertainty.

### 5.2. Endogenous Discussion

If there are endogenous variables in the explanatory variables, the estimation result of 4.1 may be biased. The per capita income of rural residents in the model may be an endogenous variable; on the one hand, the main influencing factor of consumption is income and per capita income obviously affects per capita consumption, and on the other hand, an increase in per capita consumption causes consumers to seek higher income to maintain their own consumption levels. To determine the endogeneity of this variable, a *Durbin* − *Wu* − *Hausman* test was used. The education level of rural residents is chosen as the instrumental variable, because per capita consumption does not affect the level of education, which affects the per capita income; at the same time, the change of people's education level will change people's expectation of future income, that is, it will affect the core explanatory variable, but it will have little effect on people's consumption demand, that is, it can be ignored on the explanatory variable. The least squares regression was conducted with rural per capita income as the explanatory variable and educational attainment as the explanatory variable along with other explanatory variables to obtain the residual term *μ*; the least squares regression was conducted with the residual term *μ* as the explanatory variable along with all explanatory variables in the original model and rural per capita income as the explanatory variable to obtain the coefficient *t* test of *μ* as 25.650, the concomitant probability is less than or equal to 0.001, and it is significant, so the rural per capita income is indeed an endogenous variable. To address the endogeneity of rural per capita income, the instrumental variables approach was adopted.

In order to determine whether the instrumental variables chosen above are appropriate, it is necessary to test whether the level of education directly affects per capita consumption. The test is to put the educational attainment into the random-effects regression equation in Table 4 and see if the *P* test value of the instrumental variable coefficient is greater than 0.1, which means that educational attainment does not directly affect per capita consumption and is a good instrumental variable. The *P* test value of the regression coefficient of educational attainment was found to be 0.514 (corresponding to a test value of 0.653), which means that educational attainment is a good instrumental variable.

After determining the education level as the instrumental variable, to better ensure the reliability of the regression results, 2*SLS* and dynamic *GMM* estimation methods were used to regress Equation (8) separately, and to test the variability of the results between different methods, seven different weighting methods were used in dynamic *GMM* estimation to eliminate serial correlation, the existence of heteroskedasticity between individuals, the existence of heteroskedasticity in second panel data, and the existence of temporal heteroskedasticity in individuals. The robustness of the results was verified by different estimation methods, and the results are shown in Table 6.

The regression results in Table 6 show that the estimation results for 2*SLS* and dynamics *GMM* are basically consistent, with very close coefficients for each variable, and all of them are significant at the 1% level. Compared with the results in Table 5, the relationship between each explanatory variable and the explained variable remains unchanged and positively correlated, but there is a significant change in the degree of influence. Among them, the influence of consumption in the previous period increases significantly, while the influence of income in the previous period decreases, indicating that the “ratchet effect” of rural residents' consumption is stronger; the main reason is the low level of income, easy to be affected by their own consumption habits; the influence of income uncertainty also increases significantly, indicating that rural residents' consumption may still be at a lower level; “windfall” will significantly increase the level of consumption, and “loss of income” will significantly reduce the level of consumption. After the elimination of endogenesis, the impact of urbanization and prices has been greatly weakened, indicating that urbanization may not have a relatively positive promoting effect on the income of rural residents, resulting in a failure to significantly increase the consumption level of rural residents, the reason may be that China's urbanization is more reflected in the urbanization of land and the concentration of resources in cities and towns and that rural residents do not share much in the process; most of the rural residents in China are engaged in manual labor, and their income is relatively low in the cities, which does not play an obvious role in promoting consumption, coupled with the high proportion of rural households in China that are self-sufficient, and rural residents are not price sensitive.

### 5.3. Robustness and Further Discussion

#### 5.3.1. Robustness Tests

The discussion of the endogeneity issue in Section 4.3 tests the robustness of the regression results to a certain extent. To further enhance the credibility of the results, this part tests the robustness of the estimation results by multiple means, through time period and subregional tests and by replacing the core explanatory variables, i.e., estimating Equation (9).

*(1) Robustness Tests Over Time*. To avoid possible additional autocorrelation problems associated with taking the mean value of the variables, robustness tests were conducted by taking values two years apart. As with the national regression process, after unit root tests and cointegration tests on the series of variables, 2*SLS* and dynamic *GMM* methods were used for estimation. The results of the unit root and cointegration tests show that the series of each variable in the time period are all first-order single-integer series with cointegration (specific test results omitted).

The results of the regressions by time period are homogeneous with no change in direction for each variable compared to Table 6, indicating that the municipal findings are robust. What has changed significantly in Table 7 is that the effects of urbanization rate and prices have increased significantly, and the effect of income uncertainty is no longer significant. This is due to the fact that the time length of the split-time test is only 7 years, and the urbanization process attracts a large number of rural people to work in cities in the short term, which makes the income of rural residents increase significantly and effectively stimulates the consumption of rural residents, while urbanization cannot continue to transfer a large number of rural laborers in the long term, which has a limited pull on the income of rural residents and a limited stimulation of consumption; for a short time, rural residents are not yet aware of the income. In the short term, rural residents are not aware of the impact of income uncertainty, and their psychological feeling of income uncertainty is weak, so the impact is not significant; in the short term, prices increase due to consumption inertia and the “ratchet effect,” and in order to maintain the original consumption level, rural residents' expenditure increases more, so the impact of prices in the short term is more obvious.

*(2) Robustness Tests by Region*. Similar to the analysis of the 31 provinces (municipalities directly under the central government) in China, the unit root test and cointegration test results of the variable series of different regions in East, Central, and West are consistent with the national one. To save space, only the dynamic panel 2*SLS* estimation results and the *White* *diagonal* weighted *GMM* estimation results of East, Central, and West are given below Table 8.

The regression results for East, Central, and West do not change in direction, and the relationship between the explanatory variables and the explained variables is still positive, again indicating the robustness of the findings. For East, Central, and West, the impact of prior period consumption is roughly the same, indicating that the “ratchet effect” of rural residents in East, Central, and West is basically comparable; the impact of prior period income is smaller for East and relatively larger for Central and West, because the income level of rural residents in East is much higher than that in Central and West, and rural residents in East are less dependent on prior period income. The impact of urbanization on the eastern region is very small or even negligible, and the impact is very insignificant, which is due to the high degree of urbanization in the eastern region; the impact on the consumption of rural residents has been basically released, the impact of urbanization in the western region is obviously improved compared with the eastern region, and the impact of urbanization in the central region. The impact of urbanization in the central region is the highest because the central region has a concentrated population, and the role of urbanization in stimulating consumption is strong, while the western region is subject to a special geographical environment, urbanization is slower, and the stimulating effect on consumption is not as obvious as in the central region; income uncertainty has a positive impact on both the East, Central, and Western regions, with the smallest impact in the eastern region and the largest impact in the western region, for reasons similar to those of income in the previous period, with high income in the east and a very low percentage of uncertain income. The impact on consumption is limited, and the lowest income in the West, with a relatively high proportion of uncertain income, has a significant impact on consumption relative to the east; price level has a positive impact on both the East, Middle, and West, with the smallest impact in the East and the largest impact in the West, but the difference is not significant.

#### 5.3.2. Robustness Tests for Replacing Core Explanatory Variables

To test the robustness of the empirical results from additional perspectives, the approach of replacing the core explanatory variables is tested again, using the income volatility ln*Y*_*tv*_ obtained by *HP* filtering as a proxy for income uncertainty, i.e., regression estimation of Equation (9). The previous unit root and cointegration tests provide the basis for estimating Equation (9), and the following directly employs 2*SLS* and dynamic *GMM* methods for estimation.

The results of the Tables 6 and 9 show that the explanatory variables show a positive relationship with the explanatory variables, both in terms of adjusted rates of deviation and in using income volatility to represent income uncertainty, differing only in the magnitude of the effect, again indicating that the results of Table 6 are plausible.

Combining with the test results of endogenesis, multiple regression methods, time division, region division, and substitution core explanatory variables discussed in this paper, it is fully proved that the result of Table 6 is robust and the conclusion is reliable.

#### 5.3.3. Further Discussion

In order to fully appreciate the role of the core explanatory variables on the consumption of rural residents, particularly at different levels of consumption, and also as a further test of the robustness of the estimation results, the following panel model quintiles regressions are adopted and estimated at the 10%, 30%, 50%, 70%, and 90% levels (only results where the core explanatory variables are adjusted for the rate of deviation are presented).

The test of regression coefficients for the quantile regression model shows in Table 10 (test procedure omitted) that all coefficients pass the test except ln*UR*_*t*_ when they (*τ*) are insignificant at 0-0.2.8, indicating that the results of the quantile regression are acceptable. The relationship between each explanatory variable and the explanatory variable is fully consistent with Table 6 for both the low quantile regression results and the high quantile regression results, indicating that the estimates in Table 6 are robust and reliable.

The impact of income uncertainty on rural residents' consumption is always positive during the transition from low to high levels of consumption. The impact of income uncertainty declines in the process of shifting from minimum to low consumption, indicating that rural residents do not give much thought to whether their actual income is in line with their expectations when they increase their consumption at very low levels, as the increased consumption at this point is basically spontaneous. In the shift from low to high consumption, the influence of income uncertainty tends to rise, due to the fact that during this period, rural residents have greater flexibility in consumer spending, and some commodities can be consumed or not, as confirmed by changes in the impact of price levels. The decline in the impact of income uncertainty in the shift from medium to high consumption is due to the higher income levels of the high-consumption group, which is less concerned with relatively small “windfalls” or “loss of income.”

## 6. Conclusions and Insights

In this paper, using panel data of 31 provinces across China from 2000 to 2020, we calculate the adjusted deviation rate indicating income uncertainty and obtain another variable representing income uncertainty by the *HP* filtering method, conduct a unit root test of panel data to test the smoothness of the variables, then test the cointegration relationship among the variables, and conclude that all variables are first-order single integer and have cointegration relationship. Using the *F* test and *Hausman* test to determine the random-effects model, the least squares method of panel data is applied to estimate the effects of income uncertainty, lagged one-period consumption, lagged one-period income, urbanization rate, and price level on the consumption level of rural residents, and good instrumental variables are selected based on the discussion of endogeneity issues and estimated using 2*SLS* and multiple dynamic *GMM* methods; the core explanatory variables are replaced by time period, region, and other means to test the robustness of the estimation results, further discuss the impact of income uncertainty on rural residents' consumption levels at different consumption levels using a panel quantile model, and obtain the following conclusions.

- There is a homogeneous movement between income uncertainty and rural residents' consumption, and since the proxy variables for income uncertainty used in the paper have positive and negative signs, this means that for rural residents, real income exceeding psychological income stimulates consumption and real income falling short of psychological income reduces consumption. Specifically for the East, Middle, and West, the impact is the greatest for the West and the least for the East. This is because higher real incomes make consumers more optimistic and thus more willing to spend, while lower real incomes make consumers more pessimistic and less likely to spend. The income gap in different regions of China is obvious, with the highest per capita income in the East, next in the Middle, and lowest in the West. The change of real income has different effects on different income groups and has the least effect on the high-income groups; the impact on low-income groups is greatest.
- The consumption of rural residents has a “ratchet effect,” with the consumption in the previous period moving in the same direction as the consumption in the current period, and the “ratchet effect” in the East, Middle, and West is roughly equal. Urbanization and rural consumption are in the same direction, with the highest impact in the central region, followed by the western region, and little impact in the eastern region. The price level and rural consumption move in the same direction, with slightly different effects on the East, Central, and West, but the differences are not significant. This is because the overall level of consumption of rural residents is not high, more to meet the basic needs of life, less enjoyable consumption, has obvious consumption inertia. In addition, urbanization has generally boosted the income level of rural residents, thus driving up the level of consumption. The level of urbanization in the eastern region is very high, basically over 80%, and the level of urbanization in the central region, especially in the western region, is still relatively low, about 60%, so the promotion of urbanization has little impact on the eastern region, due to the sparsity of population in the western region, the impact of urbanization is relatively limited, the central region as a population concentration of the region, and the impact of urbanization is relatively obvious.
- The quantile model indicates that income uncertainty has a greater impact on the middle- and high-consumption groups and a smaller impact on the low-income groups. The consumption of low-income groups themselves is mostly survival consumption, and whether they have more or less income has little influence on consumption. In addition to survival consumption, middle- and high-income groups also have different proportions of development consumption and enjoyment consumption, and the income change will have the obvious influence to the development consumption and the enjoyment consumption.

The policy implications of the above empirical findings are threefold: First, we should highly implement the spirit of the General Secretary's important speech on the “three rural issues,” truly realize “making farmers an attractive occupation,” and take various measures to increase the income of rural residents, continuously. We should take various measures to increase the income of rural residents, so as to obtain “unexpected benefits” and make up for the possible “income loss,” promote consumption of rural residents, and realize consumption upgrade. Second, we should pay attention to the differences in factors affecting the consumption of rural residents in the East, Central, and West and implement different policy preferences in different regions, so as to narrow the regional differences between the East, Central, and West according to local conditions. Third, on the basis of “putting the interests of farmers in the first place,” give priority to the income growth of rural low-income groups, prevent the return of poverty due to various reasons on the basis of poverty eradication, and promote the common prosperity of the majority of farmers.

## Figures and Tables

**Table 1:** Descriptive statistics of variables.

	ln*RC*_*t*_	ln*RY*_*t*_	ln*UR*_*t*_	ln*P*_*t*_	ln*EAD*_*t*_	ln*Y*_*tv*_
Average value	8.16	8.42	0.40	0.80	-0.07	0.001
Median	8.14	8.40	0.40	0.79	-0.01	-0.02
Maximum value	9.59	9.50	0.64	1.05	0.15	1.14
Minimum value	6.64	7.57	0.17	0.67	-0.73	-1.14
Standard deviation	0.65	0.43	0.10	0.09	0.18	0.34
Skewness	0.08	0.27	0.30	0.22	-2.11	0.14
Kurtosis	2.01	2.55	2.83	1.79	6.30	3.76
J-B statistic	27.32	13.71	10.65	45.00	777.30	17.78
Probability	≤0.001	≤0.001	≤0.001	≤0.001	≤0.001	≤0.001
Cumulative sum	5314.36	5482.02	259.42	518.14	-44.83	0.002
Sum of squares	270.87	118.52	7.09	5.05	20.52	74.35

**Table 2:** Unit root test results for panel data.

Variables	Method				
	*LLC* test		*ADF* test		Conclusion
	Test value	*P* value	Test value	*P* value	
ln*RC*_*t*_	1.914	0.972	7.3569	1.000	Nonstationary
ln*RY*_*t*_	0.431	0.667	63.800	0.413	Nonstationary
ln*UR*_*t*_	-1.189	0.117	51.999	0.814	Nonstationary
ln*P*_*t*_	3.610	0.999	2.491	1.000	Nonstationary
ln*EAD*_*t*_	5.429	1.000	41.725	0.978	Nonstationary
ln*Y*_*tv*_	13.692	1.000	7.910	1.000	Nonstationary
Δln*RC*_*t*_	-4.124	≤0.001^∗∗∗^	152.919	≤0.001^∗∗∗^	Stable
Δln*RY*_*t*_	-62.977	≤0.001^∗∗∗^	586.953	≤0.001^∗∗∗^	Stable
Δln*UR*_*t*_	-1.420	0.078^∗^	139.811	≤0.001^∗∗∗^	Stable
Δln*P*_*t*_	-11.519	≤0.001^∗∗∗^	215.959	≤0.001^∗∗∗^	Stable
Δln*EAD*_*t*_	-3.710	≤0.001^∗∗∗^	254.406	≤0.001^∗∗∗^	Stable
Δln*Y*_*tv*_	-2.015	0.022^∗∗^	65.791	0.347	Stable

Note: ^∗^ indicates significance at the 10% level, ^∗∗^ indicates significance at the 5% level, ^∗∗∗^ indicates significance at the 1% level, and Δ indicates first-order difference. The *ADF* test of the first-order difference series of ln*Y*_*tv*_ shows nonstationary, the *LLC* test shows stationary, so the *PP* test with the same hypothesis as *ADF* is added, and the *PP* test shows stationary (test value 78.692, *P* value = 0.075^∗^). The overall assessment is that ln*Y*_*tv*_ is a first-order smooth series.

**Table 3:** Panel cointegration tests for the variables used in Equation (8).

Variables		Panel cointegration test results				
Explained variables ln*RC*_*t*_	Explanatory variables ln*RY*_*t*_ln*EAD*_*t*_ ln*P*_*t*_ln*UR*_*t*_	Within-group statistics	*v* − *Stat* 0.312	*rho* − *Stat* 2.248	*pp* − *Stat* -2.775^∗∗∗^	*ADF* − *Stat* -3.068^∗∗∗^
		Between groups statistics		*rho* − *Stat* 3.969	*pp* − *Stat* -3.185^∗∗∗^	*ADF* − *Stat* -5.396^∗∗∗^

**Table 4:** Panel cointegration tests for the variables used in Equation (9).

Variables		Panel cointegration test results				
Explained variablesln*RC*_*t*_	Explanatory variables ln*RY*_*t*_ln*EAD*_*t*_ ln*P*_*t*_ln*UR*_*t*_	Within-group statistics	*v* − *Stat* -2.508	*rho* − *Stat* 0.838	*pp* − *Stat* -2.775^∗∗∗^	*ADF* − *Stat* -6.367^∗∗∗^
		Between groups statistics		*rho* − *Stat* 3.194	*pp* − *Stat* -6.032^∗∗∗^	*ADF* − *Stat* -2.506^∗∗∗^

Note: ^∗^ indicates significance at the 10% level, ^∗∗^ indicates significance at the 5% level, and ^∗∗∗^ indicates significance at the 1% level. All are left-tailed tests except for *v* − *Stat*, which is a right-tailed test.

**Table 5:** Fixed and random-effects estimation results for the general panel model of Equation (8).

Explanatory variables	Random-effects model		Fixed-effects model	
	Regression coefficient	*t* statistical	Regression coefficient	*t* statistical
Constant term	0.351	5.829^∗∗∗^	0.351	5.829^∗∗∗^
ln*RC*_*t*_(−1)	0.532	16.007^∗∗∗^	0.532	16.007^∗∗∗^
ln*RY*_*t*_(−1)	0.195	6.593^∗∗∗^	0.195	6.593^∗∗∗^
ln*UR*_*t*_	1.244	3.340^∗∗∗^	1.244	3.340^∗∗∗^
ln*EAD*_*t*_	0.096	4.622^∗∗∗^	0.096	4.622^∗∗∗^
ln*P*_*t*_	1.724	6.367^∗∗∗^	1.724	6.367^∗∗∗^
*Adjusted* *R*^2^ = 0.995*D* − *W* = 2.223 *F* = 24393.28*Prob*(*F*) ≤ 0.001			*Adjusted* *R*^2^ = 0.995*D* − *W* = 2.223 *F* = 3314.49*Prob*(*F*) ≤ 0.001	

Note: ^∗^ indicates significance at the 10% level, ^∗∗^ indicates significance at the 5% level, and ^∗∗∗^ indicates significance at the 1% level.

**Table 6:** Equations (8) 2*SLS* and the dynamics *GMM* of the estimation results.

Variables	Method						
	2*SLS*	*GMM*					
		2*SLS*	White cross	White period	White diagonal	Period SUR	Period weights
	(1)	(2)	(3)	(4)	(5)	(6)	(7)
ln*RC*_*t*_(−1)	0.853^∗∗∗^ (40.583)	0.853^∗∗∗^ (40.583)	0.853^∗∗∗^ (22.725)	0.851^∗∗∗^ (40.814)	0.850^∗∗∗^ (40.495)	0.852^∗∗^ (44.953)	0.853^∗∗^ (41.960)
ln*RY*_*t*_(−1)	0.109^∗∗∗^ (8.010)	0.109^∗∗∗^ (8.010)	0.111^∗∗∗^ (3.950)	0.110^∗∗∗^ (8.012)	0.110^∗∗∗^ (8.489)	0.109^∗∗∗^ (9.144)	0.109^∗∗∗^ (8.638)
ln*UR*_*t*_	0.085^∗^ (1.910)	0.085^∗^ (1.910)	0.078^∗^ (1.695)	0.089^∗∗^ (2.222)	0.087^∗^ (1.825)	0.085 ^∗∗^ (2.146)	0.086 ^∗^ (1.903)
ln*EAD*_*t*_	0.197^∗∗∗^ (6.565)	0.197^∗∗∗^ (6.565)	0.209^∗^ (1.729)	0.195^∗∗∗^ (8.370)	0.198^∗∗∗^ (5.944)	0.196^∗∗∗^ (7.619)	0.198^∗∗∗^ (5.847)
ln*P*_*t*_	0.429^∗∗∗^ (5.309)	0.429^∗∗∗^ (5.309)	0.415^∗∗∗^ (3.291)	0.435^∗∗∗^ (5.552)	0.439^∗∗∗^ (5.462)	0.432^∗∗∗^ (5.789)	0.431^∗∗∗^ (5.384)
*R* ^2^	0.99	0.99	0.99	0.99	0.99	0.99	0.99
*D* − *W*	2.149	2.149	2.147	2.145	2.143	2.147	2.148

Note: *t* test values in brackets. ^∗^ indicates significance at the 10% level, ^∗∗^ indicates significance at the 5% level, and ^∗∗∗^ indicates significance at the 1% level.

**Table 7:** Equation (8) for the time periods 2*SLS* and dynamic *GMM* estimation results.

Variables	Method						
	2*SLS*	*GMM*					
		2*SLS*	White cross	White period	White diagonal	Period SUR	Period weights
	(1)	(2)	(3)	(4)	(5)	(6)	(7)
ln*RC*_*t*_(−1)	0.536^∗∗∗^ (5.936)	0.536^∗∗∗^ (5.936)	0.538^∗∗∗^ (3.145)	0.536^∗∗∗^ (4.990)	0.536^∗∗∗^ (5.754)	0.536^∗∗∗^ (5.856)	0.536^∗∗∗^ (6.137)
ln*RY*_*t*_(−1)	0.310^∗∗∗^ (4.986)	0.310^∗∗∗^ (4.986)	0.308^∗∗^ (2.076)	0.310^∗∗∗^ (4.426)	0.310^∗∗∗^ (4.864)	0.310^∗∗∗^ (5.113)	0.310^∗∗∗^ (5.241)
ln*UR*_*t*_	0.449^∗∗∗^ (3.127)	0.449^∗∗∗^ (3.127)	0.449^∗∗^ (2.708)	0.449^∗∗∗^ (3.192)	0.449^∗∗∗^ (3.015)	0.449^∗∗∗^ (3.041)	0.449^∗∗∗^ (3.212)
ln*EAD*_*t*_	0.349 (0.917)	0.349 (0.917)	0.332 (0.293)	0.349 (0.971)	0.349 (0.883)	0.349 (1.043)	0.349 (0.979)
ln*P*_*t*_	1.504^∗∗∗^ (5.805)	1.504^∗∗∗^ (5.805)	1.503^∗∗∗^ (5.671)	1.503^∗∗∗^ (4.712)	1.504^∗∗∗^ (5.864)	1.503^∗∗∗^ (5.479)	1.504^∗∗∗^ (5.882)
*R* ^2^	0.98	0.98	0.98	0.98	0.98	0.98	0.98
*D* − *W*	1.790	1.790	1.799	1.790	1.790	1.790	1.790

Note: *t* test values in brackets. ^∗^ indicates significance at the 10% level, ^∗∗^ indicates significance at the 5% level, and ^∗∗∗^ indicates significance at the 1% level.

**Table 8:** Robustness tests for Equation (8) by region.

Region		Variables						
		ln*RC*_*t*_(−1)	ln*RY*_*t*_(−1)	ln*UR*_*t*_	ln*EAD*_*t*_	ln*P*_*t*_	*R* ^2^	*D* − *W*
East	2*SLS*	0.879^∗∗∗^ (33.134)	0.091^∗∗∗^ (4.983)	0.052 (0.918)	0.166^∗∗∗^ (3.682)	0.367^∗∗∗^ (3.275)	0.99	2.035
	*GMM*	0.890^∗∗∗^ (33.426)	0.087^∗∗∗^ (4.894)	0.007 (0.133)	0.176^∗∗∗^ (3.679)	0.320^∗∗∗^ (3.005)	0.99	2.056

Central	2*SLS*	0.777^∗∗∗^ (11.314)	0.170^∗∗∗^ (3.611)	0.415^∗∗∗^ (1.840)	0.301^∗∗^ (2.123)	0.410 (1.240)	0.99	2.277
	*GMM*	0.805^∗∗∗^ (32.733)	0.145^∗∗∗^ (8.477)	0.259^∗∗∗^ (2.662)	0.258^∗∗∗^ (5.225)	0.459^∗∗∗^ (3.498)	0.99	2.330

Western	2*SLS*	0.761^∗∗∗^ (9.969)	0.188^∗∗∗^ (3.486)	0.254^∗^ (1.917)	0.341^∗∗∗^ (4.192)	0.489^∗∗^ (2.340)	0.99	2.129
	*GMM*	0.761^∗∗∗^ (9.981)	0.188^∗∗∗^ (3.499)	0.225^∗^ (1.686)	0.337^∗∗∗^ (3.312)	0.493^∗∗^ (2.480)	0.99	2.126

Note: *t* test values in brackets. ^∗^ indicates significance at the 10% level, ^∗∗^ indicates significance at the 5% level, and ^∗∗∗^ indicates significance at the 1% level.

**Table 9:** Estimation results of Equation (9) 2*SLS* and the dynamics *GMM*.

Variables	Method						
	2*SLS*	*GMM*					
		2*SLS*	White cross	White period	White diagonal	Period SUR	Period weights
	(1)	(2)	(3)	(4)	(5)	(6)	(7)
ln*RC*_*t*_(−1)	0.581^∗∗∗^ (5.316)	0.581^∗∗∗^ (5.316)	0.495^∗∗∗^ (2.552)	0.595^∗∗∗^ (3.969)	0.581^∗∗∗^ (5.543)	0.582^∗∗∗^ (3.159)	0.578^∗∗∗^ (5.156)
ln*RY*_*t*_(−1)	0.340^∗∗∗^ (3.638)	0.340^∗∗∗^ (3.638)	0.420^∗∗^ (2.383)	0.329^∗∗∗^ (2.689)	0.340^∗∗∗^ (3.769)	0.339^∗∗^ (2.208)	0.343^∗∗∗^ (3.568)
ln*UR*_*t*_	0.162^∗∗∗^ (3.008)	0.162^∗∗∗^ (3.008)	0.157^∗∗∗^ (2.975)	0.150 (1.375)	0.158^∗∗^ (2.531)	0.161 (1.552)	0.163^∗∗∗^ (2.937)
ln*Y*_*tv*_	0.313^∗∗∗^ (3.249)	0.313^∗∗∗^ (3.249)	0.393^∗^ (1.842)	0.302^∗∗^ (2.510)	0.312^∗∗∗^ (3.279)	0.312^∗∗^ (2.070)	0.315^∗∗∗^ (3.135)
ln*P*_*t*_	0.691^∗∗∗^ (5.202)	0.691^∗∗∗^ (5.202)	0.727^∗∗∗^ (4.454)	0.675^∗∗∗^ (3.071)	0.691^∗∗∗^ (5.215)	0.688^∗∗∗^ (2.742)	0.694^∗∗∗^ (5.156)
*R* ^2^	0.99	0.99	0.99	0.99	0.99	0.99	0.99
*D* − *W*	0.983	0.983	0.763	1.020	0.985	0.986	0.977

Note: *t* test values in brackets. ^∗^ indicates significance at the 10% level, ^∗∗^ indicates significance at the 5% level, and ^∗∗∗^ indicates significance at the 1% level.

**Table 10:** Results of panel quantile estimates.

Variables	*τ* = 0.1	*τ* = 0.3	*τ* = 0.5	*τ* = 0.7	*τ* = 0.9
ln*RC*_*t*_(−1)	0.959^∗∗∗^ (49.961)	0.957^∗∗∗^ (63.430)	0.915^∗∗∗^ (54.730)	0.883^∗∗∗^ (58.546)	0.785^∗∗∗^ (31.357)
ln*RY*_*t*_(−1)	0.027^∗∗^ (2.304)	0.030^∗∗∗^ (3.486)	0.065^∗∗∗^ (6.459)	0.085^∗∗∗^ (10.048)	0.149^∗∗∗^ (10.843)
ln*UR*_*t*_	0.070^∗^ (1.923)	0.020 (0.488)	0.030 (0.704)	0.058 (1.397)	0.145^∗^ (1.878)
ln*EAD*_*t*_	0.094^∗∗∗^ (3.241)	0.061^∗∗∗^ (4.376)	0.101^∗∗∗^ (6.545)	0.112^∗∗∗^ (7.623)	0.104^∗∗∗^ (3.108)
ln*P*_*t*_	0.233^∗∗∗^ (3.587)	0.186^∗∗∗^ (2.871)	0.274^∗∗∗^ (3.706)	0.391^∗∗∗^ (5.110)	0.738^∗∗∗^ (6.005)
*R* ^2^	0.91	0.93	0.93	0.92	0.89

Note: *t* test values in brackets. ^∗^ indicates significance at the 10% level, ^∗∗^ indicates significance at the 5% level, and ^∗∗∗^ indicates significance at the 1% level.

## Data Availability

The data that support the findings of this study are available from the corresponding author upon reasonable request.
